# The Predictive Values of MMP-9, PLTs, ESR, and CRP Levels in Kawasaki Disease with Cardiovascular Injury

**DOI:** 10.1155/2022/6913315

**Published:** 2022-09-14

**Authors:** Yinan Yang, Xiaobin Hu

**Affiliations:** ^1^Department of Pediatrics, Lanzhou University Second Hospital, Lanzhou University, Lanzhou, Gansu, China; ^2^Epidemiology and Health Statistics, School of Public Health, Lanzhou University, Lanzhou, Gansu, China

## Abstract

**Objective:**

To explore the levels of matrix metalloproteinase-9 (MMP-9), platelets (PLTs), C reactive protein (CRP), and erythrocyte sedimentation rate (ESR) and their predictive values in Kawasaki disease (KD) with cardiovascular injury.

**Methods:**

128 children were diagnosed with KD in the Lanzhou University Second Hospital. 75 patients had coronary artery lesion (CAL), while 53 patients did not. The levels of MMP-9, PLTs, and CRP and ESR in the two groups were determined. The area under the curve (AUC) of the receiver-operating characteristic (ROC) curve and the Youden index (YI) were used to evaluate the efficacy of MMP-9, PLTs, ESR, and CRP for predicting CALs in KD.

**Results:**

The mean age of the patients was 2.7 ± 2.03 years (range, 2 months to 11 years). There were 87 boys (67.97%) and 41 girls (32.03%). In contrast to the NCAL group, the CAL group had obviously higher levels of MMP-9, PLTs, and CRP and an obviously higher ESR (*P* < 0.05). MMP-9 showed a linear positive correlation with ESR (*P* < 0.05) and CRP (*P* < 0.05). The AUC of the combined detection of the four indicators was 0.877, the sensitivity was 85.07% and the specificity was 78.95%.

**Conclusion:**

MMP-9, PLTs, ESR, and CRP are important indicators for a CAL in KD. The efficacy of the combined detection of MMP-9, PLTs, ESR and CRP is better than that of any single indicator for predicting a CAL in KD.

## 1. Introduction

Kawasaki disease (KD), also known as mucocutaneous lymph node syndrome, is a self-limiting disease whose major symptom is systemic arteritis. Doctor Tomisaku Kawasaki described KD for the first time in Japan in 1967 [1]. The highest incidences are seen in Japan, Korea, and Taiwan [2]. KD was also reported in China in the 1970s [3–5]. Currently, the disease has been reported worldwide [6–10]. Since the first report on KD was made 50 years ago, the etiology and pathogenic mechanism of KD remain unclear. The clinical manifestations of this disease include fever, a polymorphous rash, lymph node swelling in the neck, bilateral bulbar conjunctival congestion, alterations in the oral mucous membrane, and peripheral limb changes.

KD is pathologically characterized by the systemic inflammation of the walls of both small and medium-sized blood vessels, particularly the coronary arteries, and of multiple organs and tissues [11]. KD most frequently affects children under the age of five years [12]. Coronary artery lesions (CALs) are the most serious complication of KD and may last for many months or many years. Coronary artery dilatation and coronary artery aneurysm (CAA) are common in the acute phase, and the proportion of coronary artery stenosis gradually increases after convalescence [13, 14]. A large number of follow-up studies showed that approximately 50% of CAAs subsided within 1–2 years after onset, 80% of mild to moderate CAAs subsided within 5 years after onset [15–19], CAA diameter >5 mm may progress to stenosis, and that larger coronary artery abnormalities are associated with a greater possibility of stenosis [20]. Coronary artery abnormalities lead to potential hazards that are associated with ischemic heart disease (IHD), myocardial infarction (MI), and even sudden cardiac death (SCD) [21, 22].

Currently, CALs caused by KD have become one of the major causes of acquired heart diseases in children in Western countries and in China [23]. Studies have shown that children with KD have a higher risk of cardiovascular disease in adulthood, which is closely related to SCD in young adults and to coronary atherosclerosis in adults [17, 24]. Early exposure to high doses of intravenous immunoglobulin can reduce the incidence of CALs from 20% to 25%, and then to <5% [4].

It has been 50 years since the first report on KD was published in 1967 [12, 25]. KD has become a greater concern to an increasing number of pediatricians and cardiologists in recent years [24, 26] because KD patients show functional and structural alterations as adults due to coronary artery sequelae [28–30]. These patients may have coronary artery events in adulthood, long after the acute illness [5, 18, 31]. Therefore, the early diagnosis and treatment of KD is especially important. The purpose of this study was to find laboratory indicators with high sensitivity and specificity and to improve the early diagnosis and treatment of KD [32].

Matrix metalloproteinase-9 (MMP-9), an important member of the MMP family, may be involved in multiple inflammatory reactions. MMP-9 is considered to be very closely associated with vascular lesions in multiple diseases [33]. Studies have shown that MMP-9 plays an important role in the occurrence and development of vascular inflammation and can be used as a biochemical marker for the prediction and early diagnosis of CALs [34]. Platelets (PLTs), erythrocyte sedimentation rate (ESR), and CRP are classic inflammatory indicators in the peripheral blood for the early diagnosis of inflammatory diseases in clinical practice. Since KD is essentially a kind of vasculitis, these indicators have become increasingly meaningful in the clinical diagnosis of KD [35]. Thus, the present study aimed to examine the values of MMP-9, PLTs, ESR, and CRP for predicting CALs in KD via the combined detection of their levels.

## 2. Materials and Methods

### 2.1. Research Subjects

This study included 128 children who were diagnosed with KD based on clinical symptoms and color doppler echocardiography who were hospitalized from November 2015 to December 2018 at Lanzhou University Second Hospital. The age of the onset ranged from 2 months to 11 years old. There were 87 boys and 41 girls, with a male/female ratio of 2.12 : 1. The present research was approved by the Medical Ethics Committee of this hospital. The children's parents had signed the informed consents before the implementation of the study.

### 2.2. Diagnostic Criteria

The diagnostic criteria for the complete Kawasaki disease (CKD) were based on the 5th revised edition of the Kawasaki Disease Research Committee of Japan [36]. The diagnostic criteria for the incomplete Kawasaki disease (IKD) were based on the criteria developed by the American Heart Association (AHA) in 2004 [21]. The diagnostic criteria for CALs in KD were based on the 2015 diagnostic criteria for KD, as described in *Zhu Futang Pediatrics* (8^th^ Edition) [37].

## 3. Methods

After all the patients were admitted and their diagnosis was confirmed, 3∼5 ml of peripheral venous blood was collected and stored in an anticoagulation tube (EDTA) before 8 AM. After settling, the blood was centrifuged at 3000 r/min for 15 min to collect the upper layer of the serum. The serum MMP-9 level was detected by a double-antibody sandwich enzyme-linked immunosorbent assay (ELISA). An MMP-9 kit was purchased (Elabscience Biotechnology Co. Ltd., Wuhan, China), and the assay was executed in strict accordance with the instructions of the kit. Then, MMP-9 levels were detected by using an Infinite F200 Multifunctional Microplate Reader (Tecan, Sweden). The ESR was determined by the Westergren method, and the levels of PLTs and CRP were detected by using an ADVIA70 Automatic Hematology Analyzer (Bayer, Germany). The levels of albumin (ALB) were detected by using an ADVIA Chemistry XPT Fully Automatic Biochemical Analyzer (Siemens, Germany).

### 3.1. Statistical Methods

The data obtained were analyzed by SPSS 22.0 software and GraphPad Prism 8.0 software. Measurement data with a normal distribution are expressed as the mean ± the standard deviation (SD). Group comparisons were made by two independent-sample*t* tests. The categorical data was expressed as *n* (%), and the comparison of categorical data were performed by the chi-square test. Correlations between two variables were analyzed by the Spearman correlation analysis. The area under the curve (AUC) of the receiver-operating characteristic (ROC) curve and the Youden index (YI) were used to evaluate the efficacy of MMP-9, PLTs, ESR, and CRP for predicting CALs in KD. As the AUC gets closer to 1, the diagnostic efficacy increases. (*P* < 0.05) was considered statistically significant.

## 4. Results

The mean age of the patients was 2.7 ± 2.03 years (range, 2 months to 11 years). There were 87 boys (67.97%) and 41 girls (32.03%), with a male/female ratio of 2.12 : 1. Among the patients, the incidence of KD in infancy was obviously higher than that in other age groups, and 55 (43.0%) patients were under the age of one year. The details of the demographic data of the study participants are shown in Table 1 and Figure 1. All patients were treated with the regular medications, and 75 (58.59%) had a CAL. According to the clinical manifestations and coronary artery injury status, the patients were divided into the CKD group and the IKD group. A total of 56 patients had CKD (43.8%), and 72 (56.2%) patients had IDK. A comparison of the sex and age characteristics between the CKD and IKD groups is shown in Table 2. There was no significant difference in the age and gender between the two groups (*P* > 0.05).

Of the 56 patients with CKD, 27 patients (48.21%) had a CAL and 29 patients (51.69%) had NCALs (no coronary artery lesions). Among the 72 patients with IKD, 48 patients (66.67%) had a CAL and 24 patients (33.33%) had NCALs. The difference between the two groups was statistically significant (*X*^2^ = 4.421, *P*=0.036, *P* < 0.05), indicating that the incidence of CALs was significantly higher in the IDK group than in the CKD group (Figure 2).

### 4.1. Comparisons of the Levels of MMP-9, PLTs, CRP, and ALB and ESR between the CAL Group and the NCAL Group

The statistical analysis of laboratory indicators in the CAL group and the NCAL group showed that the levels of MMP-9, PLTs, and CRP and the ESR were much higher in the CAL group, and ALB was lower in the NCAL group; these differences were statistically significant (*P* < 0.01). Compared with IKD, CKD had a significantly higher concentration of MMP-9, and this difference was statistically significant (*P* < 0.05) (Figure 3).

### 4.2. Correlations of MMP-9 with PLTs, ESR, and CRP

Spearman correlation analysis suggested that MMP-9 showed a linear positive correlation with the ESR (*r* = 0.224, *P* < 0.05) and CRP (*r* = 0.352, *P* < 0.05) (Figure 4); the PLT levels were not obviously correlated with MMP-9.

### 4.3. The Results of the ROC Curve Analysis for MMP-9, PLTs, ESR, and CRP

The AUCs of the ROC curves for MMP-9, PLTs, ESR, and CRP were 0.636 (95% CI 0.532∼0.741), 0.681 (95% CI 0.589∼0.772), 0.762 (95% CI 0.671∼0.853), and 0.657 (95% CI 0.564∼0.750), respectively, (ESR˃PLT˃CRP˃MMP-9). The YIs of MMP-9, PLTs, te ESR, and CRP were 0.372, 0.408, 0.530, and 0.330, respectively, (ESR˃PLT˃MMP-9˃CRP). From the perspective of the best diagnostic cut-off value, when MMP-9 was set to 1120.74 ng/mL, the sensitivity and specificity for CALs and NCALs in KD were 58.21% and 78.95%, respectively. When the PLT cut-off was set to 424.5 × 10^9^/L, the sensitivity and specificity for CALs and NCALs in KD were 42.67% and 98.11%, respectively. When the ESR cut-off was set to 74.5 mm/h, the sensitivity and specificity for CALs and NCALs in KD were 81.3% and 71.7%, respectively. When the CRP cut-off was set to was 82.5 mg/L, the sensitivity and specificity for CALs and NCALs in KD patients were 38.67% and 94.34%, respectively (Table 3).

To make up for the limitation of a single diagnostic index, we determined the optimal cut-off values of MMP-9, PLTs, ESR, and CRP by using the ROC curves. The four values were converted into different combined indicators by the multiple factor logistic regression, and the regression equation of the combined indicators for diagnosis was expressed as log(*P*) = 0.0001^*∗*^MMP-9−0.005^*∗*^PLT−0.036^*∗*^ ESR−0.019^*∗*^CRP−4.791. The predicative factor *P*=1/(1 +e – (0.001 ^*∗*^ MMP-9−0.005 ^*∗*^ PLT−0.036^*∗*^ ESR−0.019^*∗*^ CRP−4.791)) was obtained after performing a conversion. A ROC curve was drawn with the predicative factor *P* as the indicator for the analysis of the combined factors for diagnosis. The AUC of the combined detection of the four indicators was 0.877, the SD was 0.034, the sensitivity was 85.07%, and the specificity was 78.95%. The AUC for the combined factor diagnosis yielded the following results: compared with the AUC of MMP-9 for diagnosis, *Z* = 3.84 and *P* < 0.05; compared with the AUC of PLTs for diagnosis, *Z* = 3.40 and P˂0.05; compared with the AUC of the ESR for diagnosis, *Z* = 2.00 and *P* < 0.05; and compared with the AUC of CRP for diagnosis, *Z* = 3.76 and *P* < 0.05; these differences were statistically significant (*P* < 0.05). These results show that the AUC, sensitivity, and specificity of the combined diagnosis with four indicators were superior to those of the single indicators. Thus, the combination of the four indicators was considered the most effective way to distinguish CALs and NCALs, as the efficacy was superior to that of the single indicators, and the rate of missed diagnoses and misdiagnoses was lower (Figure 5).

## 5. Discussion

KD, a kind of disease whose major symptom is vascular inflammation, mostly occurs in children. It is difficult to distinguish these conditions from infectious febrile diseases in the absence of specific laboratory diagnostic indictors [38, 39]. Thus, the early diagnosis and prediction of CALs in KD is of great significance for understanding the development, progression, and severity of this illness [40].

MMPs are zinc-dependent proteases that were first discovered in 1962 that play an important role in the cardiovascular disease [41–45]. In the MMP family, MMP-9 is the member that is most closely associated with vascular lesions [46–50], including acute MI, atherosclerosis, heart failure, and aortic aneurysm [51, 52]. MMP-9 activity contributes to the decomposition of elastin, and blocking this activity can decrease coronary artery inflammation in KD animals [53, 54]. In our study, we found that MMP-9 was not only upregulated in KD but was also significantly correlated with CALs, which is consistent with a report by Kuo et al. [55].

Elevations in MMP-9, PLTs, ESR, and CRP in children should be given adequate attention in clinical practice, thus avoiding the occurrence or further development of CALs. Lai [56] found that serum MMP-9 was positively correlated with serum CRP and the ESR in CALs based on partial correlation analysis, which may be explained by the fact that the ESR is mainly affected by changes in immunoglobulins and fibrinogens in the blood. MMP-9 may be activated by neutrophil elastase, plasminogen activators, and fibrin plasmin in the inflammatory response, further accelerating ECM degradation and leading to the destruction of the vascular wall [57]. Thus, there is a mechanism through which the ESR and MMP-9 can simultaneously increase, leading to the positive correlation of these factors. CRP is involved in the entire process of the inflammatory response, as it activates complement proteins and increases the ability of monocytes to release [58], while monocytes are stimulated by IL-1*β* to produce prostaglandin E2 and, therefore, to generate MMP-9 [59]; in addition, CRP is synthesized and secreted by hepatocytes that are stimulated by cytokines, such as IL-6 and IL-1*β*, revealing the interaction between CRP and MMP-9. CRP is able to induce an increase in the MMP-9 expression. Hence, there is a certain correlation between CRP and MMP-9.

The combined detection of MMP-9, PLTs, ESR, and CRP is superior to the detection of any single indicator for predicting CALs in KD. The etiology and pathogenesis of KD are not fully understood, and clinicians lack specific laboratory criteria for diagnosis, making it difficult to make an early diagnosis of KD. Moreover, many KD patients come to the hospital for medical treatment because of a fever of an unknown cause and have no typical clinical characteristics. The progressive aggravation of inflammation leads to the persistence of a vascular inflammatory response that increases in severity, thus causing CALs [60]. Therefore, KD should be considered in patients with a fever of an unknown origin in the acute stage if the index of the appeal is abnormally increased.

Because CAL in KD usually appears two weeks after the onset of the disease, it is more difficult to make an early diagnosis of IKD [61]. PLTs, ESR, CRP, and other inflammatory indicators have been increasingly useful for the clinical diagnosis of KD and have been widely recognized by the majority of clinicians. However, reports comparing the efficacy of these indicators in the early diagnosis and prediction of CALs are rare. The detection results of MMP-9, PLTs, ESR, and CRP in this study showed that the ESR has good sensitivity and specificity, while PLTs, CRP, and MMP-9 have lower sensitivity and higher specificity, and thus have limited diagnostic values. After combining the four indicators into a singer diagnostic indicator by logistic stepwise regression, the ROC analysis suggested that the sensitivity and specificity has improved. Therefore, combined detection was considered to have a higher efficacy for predicting CALs in KD and to perform better than single-indicator detection, suggesting that both missed diagnoses and the misdiagnosis rate would be reduced.

There are some limitations in this study. This study was a single center clinical study, with limited sample size and less variables. In the future, large sample and long follow-up studies are needed to verify the role of MMP-9, PLTs, ESR, and CRP levels in Kawasaki disease with cardiovascular injury.

## 6. Conclusions

In conclusion, the combined detection of MMP-9, PLTs, ESR, and CRP is of great significance for predicting CALs in children with KD and provides a theoretical basis for clinicians to achieve the early diagnosis of KD.

## Figures and Tables

**Figure 1:** Age composition ratio of children with KD.

**Figure 2:** Comparison of the incidence rate of CAL between CKD and IKD.

**Figure 3:** The CAL and NCAL groups regarding the serum levels of MMP-9, PLTs, CRP, ESR, and ALB and the concentration of MMP-9 in CKD and IKD. The level of statistical significance was set at *P* < 0.05.

**Figure 4:** MMP-9 showed a linear positive correction with the (a) ESP (*r* = 0.224, *P* < 0.05) and the (b) CRP (*r* = 0.352, *P* < 0.05).

**Figure 5:** The ROC curve analysis for MMP-9, PLTs, EST, and CEP.

**Table 1:** Age and sex composition at onset in KD (*n*%).

Age (y)	Male (*n*%)	Female (*n*%)	Total (*n*%)
≤1 y	39 (44.8%)	16 (39.0%)	55 (43.0%)
1∼3 y	31 (35.6%)	13 (31.7%)	44 (34.4%)
>3 y	17 (19.5%)	12 (29.3%)	29 (22.7%)
Total	87 (100.0%)	41 (100%)	128 (100.0%)

**Table 2:** Comparison of general characteristics between CKD and IKD.

Items	CKD	IKD	*X * ^2^	*P* value
Sex				
Male	37 (66.1%)	50 (69.4%)	0.165	0.685
Female	19 (33.9%)	22 (30.6%)		

Age (y)				
≤1 y	24 (42.9%)	31 (43.1%)	0.001	0.982
1∼3 y	23 (41.1%)	21 (29.2%)	3.440	0.064
>3 y	9 (16.1%)	20 (27.8%)	2.463	0.117

Total	56 (100%)	72 (100.0%)	3.204	0.201

*Note. P* < 0.05 was considered statistically significant.

**Table 3:** Evaluation of the detection indicators (PLTs, ESR, CRP, and MMP-9) for predicting CALs.

	AUC	SE	AUC (95% CI)	Cut-off value	Youde *n* index	Sensitivity (%)	Specificity (%)	*P*
PLT	0.681	0.047	0.589∼0.772	424.5	0.408	42.67	98.11	0.001
ESR	0.762	0.047	0.671∼0.853	74.5	0.530	81.30	71.70	0.000
CRP	0.657	0.048	0.564∼0.750	82.5	0.330	38.67	94.34	0.003
MMP-9	0.636	0.053	0.532∼0.741	1120.74	0.372	58.21	78.95	0.021

*Note. P* < 0.05 was considered statistically significant.

## Data Availability

The data used to support the findings of this study are available from the corresponding author upon request.
